# Efficacy of Neoadjuvant Chemotherapy with Epirubicin and Cyclophosphamide and Weekly Paclitaxel and Trastuzumab in Human Epidermal Growth Factor Receptor 2–Positive Breast Carcinoma: A Real-World Study

**DOI:** 10.1155/2020/3208391

**Published:** 2020-05-05

**Authors:** Mengmeng Zhang, Ling Li, Shiyong Zhang, Wenlong Zhu, Senguo Yang, Guangsheng Di, Xiaoxia Ma, Haisong Yang

**Affiliations:** ^1^Department of Breast Surgery, The Affiliated Hospital of Guizhou Medical University, Guizhou 550004, China; ^2^Department of Neurology, 925 Hospital of PLA Joint Logistics Support Force, Guizhou 550009, China

## Abstract

**Background:**

Trastuzumab has been introduced a decade ago and demonstrated improvement in the prognosis in patients with human epidermal growth factor receptor 2- (HER2-) positive (+) breast carcinoma (BC). This study is aimed at evaluating the efficacy of epirubicin/cyclophosphamide with weekly paclitaxel-trastuzumab as neoadjuvant chemotherapies in HER2+ BC patients.

**Methods:**

A total of 234 HER2+ BC patients were given neoadjuvant chemotherapy (NAC) between 2010 and 2016. The primary endpoints were pathologic complete response (pCR) and disease-free survival (DFS). Univariate and multivariate analyses of clinical and pathological factors associated with pCR and DFS were conducted.

**Results:**

The pCR (30.4% vs. 14.8%; *P* = 0.004) and DFS (*P* = 0.036) showed significant differences between patients administered with neoadjuvant trastuzumab therapy and those who did not. Multivariate logistic regression analysis showed that neoadjuvant trastuzumab treatment was regarded as an independent predictor of pCR. Patients with pCR had prolonged DFS (*P* = 0.025). In patients who did not achieve pCR (non-pCR), those who received trastuzumab had more prolonged DFS (*P* = 0.046). The luminal B/HER2+ subtypes had prolonged DFS when compared with nonluminal B/HER2+ subtypes (*P* = 0.010). The luminal B/HER2+ subgroup also showed improved DFS in non-pCR patients (*P* = 0.010). In the subgroup of non-pCR, the luminal B/HER2+ subgroup administered with trastuzumab showed no superior DFS (*P* = 0.168). However, a positive result was observed in patients without trastuzumab (*P* = 0.039). Multivariate analysis showed cT stage (*P* = 0.006) and tumor grade (*P* = 0.041), considering them as significant prognostic factors of DFS.

**Conclusions:**

HER2+ BC patients showed improvement in pCR and DFS after neoadjuvant trastuzumab treatment. Patients without pCR had prolonged DFS after trastuzumab maintenance. Although the prognosis of luminal B/HER2+ BC showed favorable outcomes in the non-pCR subgroup, those receiving trastuzumab showed no survival advantage.

## 1. Introduction

Breast carcinoma (BC) is the most commonly encountered malignancy in women and the leading cause of mortality in female patients [1]. The human epidermal growth factor receptor 2 (HER2) is overexpressed in 25% to 30% of patients with BC, and this is associated with elevated malignancy potential [2, 3]. Trastuzumab, a humanized monoclonal antibody that targets HER2 by binding to its extracellular domain as a single agent, demonstrated modest antitumor activities. It is used for treating both metastatic and early-stage HER2+ BC with high efficacy [4–6]. Randomized studies reported similar survival benefits for particular treatment regimens, regardless of whether the treatment is preoperatively or postoperatively administered. Neoadjuvant chemotherapy (NAC) for early and locally advanced BC is broadly employed to downstage the primary lesion, allowing a higher rate of breast preservation [7, 8]. In addition, it can be used for testing chemosensitivity in vivo, making it possible to assess the efficacy of early systemic therapy and to stop ineffective treatment. The achievement of pathologic complete response (pCR) upon NAC is considered an important surrogate marker to improve the long-term outcomes [8, 9]. It is hypothesized that a regimen that produces higher pCR rates in a neoadjuvant systemic therapy setting also ensues higher rates of long-term cure. Recently, phase II and III clinical studies have intensely assessed the combination of trastuzumab and NAC as neoadjuvant systemic therapy for early and locally advanced HER2+ BC, respectively [10–12]. Also, recent studies showed that NAC when combined with trastuzumab assists in achieving significantly higher pCR rates than NAC alone [10, 11, 13]. Trastuzumab-based therapy has been used over the past decade and demonstrated a favorable impact on survival when compared with the same chemotherapy alone as therapy [14]. For HER2+ BC patients who require neoadjuvant therapy, trastuzumab is generally added to chemotherapy, and the patient receives adjuvant trastuzumab for 1 year.

However, whether the results of randomized controlled trials (RCTs) are applicable to the real-world cases is one of the major issues. The present work is aimed at assessing NAC with epirubicin/cyclophosphamide (EC) and paclitaxel-trastuzumab (PH) in HER2+ BC patients. The study also explored whether the effectiveness of neoadjuvant trastuzumab in association with NAC in the real-world treatment of patients with HER2+ BC was comparable to that observed in RCTs.

## 2. Materials and Methods

### 2.1. Patient Population

In this study, 234 cases with operable or locally advanced HER2+ BC who underwent treatment at our hospital between 2010 and 2016 were analyzed. All patients underwent a core biopsy before receiving NAC, followed by surgery or radiotherapy. Before initiating the therapy, all patients underwent staging evaluation, which included a complete history check, physical examination, computed tomography (CT) scan of the chest and liver, and bone scan. Mammography of both breasts was performed, and additional breast and axillary assessment of the tumor site was done by ultrasound. This trial had approval from the Research and Ethics Committee of our hospital, and informed consent was obtained from all patients.

### 2.2. Treatments

All patients were confirmed with the diagnosis of invasive BC by biopsy before NAC, including breast ultrasonography, breast mammography, and breast magnetic resonance imaging (MRI) to confirm the tumor size; fine needle aspiration was performed to assess metastasis to axillary lymph nodes and chest ultrasonography, abdominal CT, and whole-body bone scan to exclude distant metastases. Patient treatment was based on the National Comprehensive Cancer Network guidelines. Furthermore, 92 patients received dose-dense epirubicin/cyclophosphamide and paclitaxel-trastuzumab (EC-PH) and 142 were administered with dose-dense EC-P NAC. EC-PH consisted of four cycles of EC (epirubicin/cyclophosphamide (90/600 mg/m^2^)) on day 1 treatment, administered at 2-week intervals, and paclitaxel (80 mg/m^2^) once a week for 12 weeks. Trastuzumab 4 mg/kg (loading dose) was administered on day 1 and 2 mg/kg per week for 12 weeks (NAC duration). Also, 92 patients completed trastuzumab therapy for a year. The patients underwent surgery at 1–4 weeks upon NAC completion. Surgical intervention included breast-conserving operation, mastectomy and sentinel node biopsy, or axillary lymph node dissection. Radiation therapy was administered in case of breast-conserving surgery or locally advanced disease. Patients with hormone receptor-positive (HR+) cancer received adjuvant endocrine therapy for 5 years.

### 2.3. Pathological Assessment

Immunohistochemical (IHC) assessment of human epidermal growth factor receptor 2 (HER2), estrogen receptor (ER), and progesterone receptor (PR) was conducted on pretreatment biopsies and surgical specimens by pathologists. Through IHC detection, HER23+ was considered positive, and 0-1+ was considered negative; 2+ required verification through fluorescence in situ hybridization (FISH), in which 2.2 gene copies (per FISH) were considered positive for *HER2* amplification. Nuclear staining ≥ 1% of ER or PR was deemed to be positive. For Ki-67, the positive cells demonstrated light yellow to brown nuclei under 400x light microscopy in 10 randomly selected fields. A total of 500 cells were counted in each field, and the ratio of Ki-67-positive cells to total cells was calculated. A pCR was defined as the absence of invasive residual breast tumor or invasive lesion in ipsilateral axillary nodes (ypT0 ypN0).

### 2.4. Follow-Up

From day 1 after surgery, all patients were followed up till March 2018, with the follow-up information obtained through outpatient interviews or telephone calls. Disease-free survival (DFS) was determined from day 1 after surgery to the first local relapse.

### 2.5. Statistical Analysis

The association of clinical characteristics with pCR was determined by Pearson's *χ*^2^ or Fisher's exact test. Univariate analysis was performed, and parameters showing significant associations entered the multivariate logistic models. Multivariate analysis used an unconditional stepwise logistic regression approach. Univariate/multivariate survival analyses were performed using the Cox regression model. The interactions between significant investigation variables were considered when developing the multivariate model. DFS estimation was carried out by Kaplan–Meier analysis, and the log-rank test was used to compare the groups. *P* < 0.05 was considered to be statistically significant. All statistical analyses were performed using SPSS Statistic software 19.

## 3. Results

### 3.1. Clinical Characteristics and Response to NAC

From April 2011 to August 2017, 234 patients with HER2+ BC who underwent surgery were given neoadjuvant trastuzumab combined with dose-dense EC-P. The median age of the patients was 50 years, ranging from 27 to 75 years. A total of 160 patients had T1–T2 tumors (69.2%), and 108 had lymph node metastasis (46.2%). Associations of baseline patient features and therapeutic indexes with pCR in univariate analysis are reported in Table 1. All cases had highly proliferative invasive ductal carcinoma (in which 46.6% showing Ki‐67 > 30%). Tumor grades were 1–2 in 53 (22.6%) and 3 in 181 (77.4%) cases. The luminal B/HER2+ (HER2+/ER+ and/or PR+) and nonluminal B/HER2+ (HER2+/ER– and PR–) subtypes were involved in 127 (54.3%) and 107 (45.7%) patients, respectively. The residual invasive breast lesions were found in 185 (79.1%) patients and residual noninvasive tumors in 49 (20.9%) patients. The pCR rate was increased in patients who were given neoadjuvant trastuzumab therapy (*P* < 0.05) (Table 1). Multivariate logistic regression analysis revealed that the use of trastuzumab independently predicted pCR (Table 2).

### 3.2. Patient Survival

The median follow-up was 32.9 months (range, 5–82 months), and the mean DFS was 32 months. In this study, 25/234 (10.7%) cases showed local relapse or distant metastases. In Kaplan–Meier analysis, survival showed marked differences between cases administered with trastuzumab and the remaining patients (*P* = 0.036, Figure 1). Multivariate logistic regression analysis revealed neoadjuvant trastuzumab administration (*P* = 0.004) as an independent predictive factor for pCR (*P* = 0.004, Table 2). Meanwhile, cases with pCR had prolonged DFS (*P* = 0.025, Figure 2). Among those who did not achieve pCR, patients administered with trastuzumab more likely showed a prolonged DFS (*P* = 0.046, Figure 3). However, a positive result was not observed in patients with pCR (Figure 4). Moreover, patients with luminal B/HER2+ had improved DFS (*P* = 0.010) than those with nonluminal B/HER2+ (Figure 5). The luminal B/HER2+ subtype also showed improvement in the DFS rates in non-pCR cases (*P* = 0.010, Figure 6). In subgroup analyses, patients with luminal B/HER2+ with trastuzumab administration showed no prolonged DFS in non-pCR cases (*P* = 0.168, Figure 7). However, a positive result was observed in patients without trastuzumab (*P* = 0.039, Figure 8). Multivariate analysis revealed cT stage (hazard ratio = 3.80, 95% CI 1.46–9.89; *P* = 0.006) and tumor grade (hazard ratio = 5.17, 95% CI 1.07–24.96; *P* = 0.041) as independent predictive factors for DFS in patients with BC (Table 3).

## 4. Discussion

Recent studies have focused on the relative value of RCTs to help make a routine clinical decision, as they are the major endpoints of comparative effectiveness research [15, 16]. Although findings of RCTs largely determine the comparison among treatment groups, case selection criteria and the rigidity of protocols do not allow changes easily in dose and toxicity management, making these findings not generalizable to the patient level [17]. Whether the results of these RCTs are applicable to real-world cases and whether patients can afford these drugs for some special reasons are major issues. Due to economic reasons, especially in resource-limited regions, many patients with HER2+ less likely received trastuzumab-containing treatment. In 2017, the cost of trastuzumab was substantially reduced in China, making it feasible for most of the patients to afford the drug. Accordingly, observational retrospective trials are considered important sources of data on the effectiveness of alternative therapies based on patient and tumor properties. Therefore, the present work is aimed at reporting the effectiveness of neoadjuvant trastuzumab with dose-dense EC-P in 234 cases with operable or locally advanced HER2+ BC. This novel retrospective study compared the effectiveness of EC-PH and EC-P in HER2+ BC patients. The results showed that (1) pCR was achieved in 30.4% and 14.8% of patients with and without neoadjuvant trastuzumab treatment, respectively; (2) patients with pCR had prolonged DFS; (3) neoadjuvant trastuzumab treatment independently predicted pCR and showed association with improved DFS in all patients and the non-pCR subgroup; (4) the luminal B/HER2+ subtype showed superior DFS in all patients and the non-pCR subgroup; (5) in the non-pCR subgroup, the luminal B/HER2+ subtype without neoadjuvant trastuzumab treatment showed superior DFS; and (6) cT stage and tumor grade were considered independent prognostic factors of DFS.

As expected, the results of this study confirmed that administration of trastuzumab and NAC resulted in elevated pCR rate (30.4%) when compared with the NAC-alone group (14.8%). The previously published pCR rates for NAC and trastuzumab ranged between 32% and 66% [10, 11, 18]. The reasons for the lower rate in this study might be due to its retrospective design and small sample size. In addition, there were more cases with luminal B/HER2+ than the nonluminal B/HER2+ counterpart. Multiple clinical studies have reported marked elevation in the pCR rate in the nonluminal B/HER2+ molecular subtype when compared with the luminal B/HER2+ molecular subtype [19–21]. More importantly, multivariate analysis also revealed the use of trastuzumab as an independent predictor of pCR. Therefore, trastuzumab plus NAC increased the pCR rate. Recently, many pivotal RCTs have confirmed the efficacy and safety of trastuzumab/NAC combination therapy in early and locally advanced HER2+ BC patients [10–12]. This study also revealed that the patients who were treated with trastuzumab plus NAC had prolonged DFS. These results confirmed that the eligibility criteria and treatment outcomes of clinical trials could be translated to the real-world setting.

The most recent view is that luminal B/HER2+ BC represents a distinct subgroup with lower chemotherapy sensitivity and better outcomes when compared with HR-/HER2+ disease [19, 22–24]. In the present study, DFS in the luminal B/HER2+ subtype was better than that in the nonluminal/HER2+ subtype. Moreover, positive results were observed in the non-pCR subgroup. This was due to the use of adjuvant endocrine therapy for patients with the luminal B/HER2+ subtype, which reduced the risk of recurrence. In subgroup analysis, superior DFS was observed in patients with the luminal B/HER2+ subtype without trastuzumab who did not achieve pCR. However, a negative result was observed in patients who had trastuzumab. The role of hormone receptor (HR) status in predicting pCR and prognosis upon trastuzumab-containing NAC administration is subjected to debate, although most of the trials reported positive results. Based on the previous reports, the absence of HR represents a critical predictive factor in pCR and a reliable prognostic index [20–24]. However, a crosstalk is believed to occur between the HER2 and ER pathways in ER+/HER2+ patients, while estrogen-independent ER signaling dominates the classical estrogen-dependent ER signaling pathway [25, 26]. The fact that the upregulation of ER expression and/or activity functions as an escape mechanism, leading to resistance to anti-HER2 treatment in HER2+ and HR+ BC patients [27]. Preclinical studies have shown that ER+ and HER2+ BC cell lines are initially sensitive to lapatinib. After gaining resistance to lapatinib, ER signaling showed significant enhancement, and the resistance can be prevented by simultaneous inhibition of HER2 and ER signals [28, 29]. Researchers have found that the ER functions play a key role in escaping/survival pathway of HER2+/ER+ cells under sustained HER2 inhibition and that a dynamic transition between HER2 and ER activity plays a role in resistance to regimens containing lapatinib [30]. In addition, recent findings have revealed that PIK3CA-mutated HER2+ BC patients less likely achieved pCR and prolonged DFS upon neoadjuvant anthracycline-taxane chemotherapy when combined with anti-HER2 treatment, and this might explain such discrepancy [31, 32]. Activation of the PI3K/AKT/mTOR signaling pathway is related to oncogenesis and tumor progression and resistance to standard anticancer therapies [33, 34]. The PIK3CA gene that regulates PI3K is one of the most frequently mutated genes in human cancers. Abnormal activation of the PI3K pathway is frequently observed in BC, resulting in uncontrolled tumor cell growth and drug resistance [35]. HER2+ BC carrying PIK3CA mutations is particularly dependent on the PI3K signaling pathway, and it has been shown that activation of this pathway plays a key role in developing resistance to trastuzumab [33, 36].

Whether pCR represents a surrogate marker of DFS and overall survival (OS) in HER2+ BC patients remains to be a largely controversial topic. The present study revealed that patients who achieved pCR had prolonged DFS. Meta-analysis of 6377 cases with primary BC administered with neoadjuvant anthracycline-taxane in 7 randomized studies revealed pCR as a valid substitute of DFS and OS in HER2+ subtypes [37]. In addition, three multicenter retrospective studies on HER2+ BC who underwent treatment with NAC and trastuzumab showed pCR as a surrogate marker for DFS in HR-BC, but the results of the HR+ group were negative [9, 38, 39]. However, researchers confirmed the level of evidence available for supporting a relationship between pCR and OS [40, 41]. Therefore, pCR still cannot be used as a surrogate marker for long-term survival. Subgroup analysis of the present data revealed that trastuzumab use in cases who achieved pCR did not result in favorable survival outcomes. However, our study found that patients who underwent treatment with trastuzumab plus NAC had good DFS for non-pCR responders, indicating that patients who did not achieve pCR should be treated with trastuzumab. To date, phase II and III trials have not been conducted to explore trastuzumab use following trastuzumab plus NAC administration preoperatively in cases who did not achieve pCR. The efficacy of anti-HER2 agents in non-pCR responders also remained controversial [42]. The present study results revealed that these patients gained benefits from using trastuzumab maintenance, although they are less likely to respond to trastuzumab plus NAC.

Multivariate analysis revealed cT stage and tumor grade as significant independent prognostic factors of pCR, which was consistent with the previous studies [9, 39]. The present study was limited due to its relatively small sample size, short follow-up period, and single-institution design. These patients should be followed up in the future to observe the long-term outcomes, and sample size should be enlarged to confirm the current results.

In conclusion, trastuzumab improved the prognosis of patients with HER2+ BC. NAC plus trastuzumab resulted in elevated pCR rate in HER2+ BC patients. The non-pCR cases upon neoadjuvant anti-HER2 treatment plus chemotherapy followed by trastuzumab maintenance had better long-term outcomes. Although the prognosis of the luminal B/HER2+ subtype demonstrated favorable outcomes in the non-pCR subgroup, luminal B/HER2+ BC patients receiving trastuzumab showed no survival advantage. Hence, more patients and long-term follow-up time are needed for further study. Neoadjuvant treatment with EC-PH might be a suitable alternative regimen for Chinese women who require anthracycline therapy.

## Figures and Tables

**Figure 1:** Association of trastuzumab use with DFS.

**Figure 2:** DFS in patients with pCR and non-pCR.

**Figure 3:** Association of trastuzumab use with DFS in non-pCR patients.

**Figure 4:** Association of trastuzumab use with DFS in pCR patients.

**Figure 5:** DFS curves in luminal B/HER2+ and nonluminal B/HER2+ patients.

**Figure 6:** DFS curves of luminal B/HER2+ and nonluminal B/HER2+ patients in non-pCR patients.

**Figure 7:** DFS curves of luminal B/HER2+ and nonluminal B/HER2+ patients in non-pCR patients administered with trastuzumab.

**Figure 8:** DFS curves of luminal B/HER2+ and nonluminal B/HER2+ patients in non-pCR patients without trastuzumab use.

**Table 1:** Associations of clinical characteristics with pCR in univariate analysis.

	Non-pCR (*n* = 185)		pCR (*n* = 49)		*P* value
	*n*	%	*n*	%	
Age (year)					0.182
≤35	24	13.0	3	6.1	
>35	161	87.0	46	93.9	
Menopausal status					0.527
Premenopausal	100	54.1	24	49.0	
Postmenopausal	85	45.9	25	51.0	
cT stage					0.389
cT1–2	124	67.0	36	73.5	
cT3–4	61	33.0	13	26.5	
cN stage					0.07
cN0	94	50.8	32	65.3	
cN1–3	91	49.2	17	34.7	
Grade					0.729
G1–2	41	22.2	12	24.5	
G3	144	77.8	37	75.5	
ER					0.472
Positive	105	56.8	25	51.0	
Negative	80	43.2	24	49.0	
PR					0.949
Positive	84	45.4	22	44.9	
Negative	101	54.6	27	55.1	
HR					0.854
Positive	82	44.3	21	42.9	
Negative	103	55.7	28	57.1	
Ki-67					0.791
>30%	87	47.0	22	44.9	
≤30%	98	53.0	27	55.1	
Molecular subtype					0.607
Luminal B/HER2+	102	55.1	25	51.0	
Nonluminal/HER2+	83	44.9	24	49.0	
Trastuzumab					*0.004*
Yes	64	34.6	28	57.1	
No	121	65.4	21	42.9	

**Table 2:** Predictive factors of pCR according to the multivariate logistic regression model.

	Univariate			Multivariate		
	OR	95% CI	*P* value	OR	95% CI	*P* value
Age (year)			0.193			0.189
≤35	1.000			1.000		
>35	2.286	0.659–7.931		2.438	0.645–9.209	
Menopausal status			0.527			0.727
Premenopausal	1.000			1.000		
Postmenopausal	1.225	0.652–2.303		1.130	0.570–2.237	
cT stage			0.39			0.900
cT1–2	1.000			1.000		
cT3–4	0.734	0.363–1.485		0.951	0.436–2.075	
cN stage			0.073			0.324
cN0	1.000			1.000		
cN1–3	0.549	0.285–1.057		0.698	0.342–1.425	
Grade			0.729			0.453
G1–2	1.000			1.000		
G3	0.878	0.420–1.836		0.738	0.334–1.631	
ER			0.473			0.311
Positive	1.000			1.000		
Negative	1.260	0.670–2.368		2.415	0.439–13.279	
PR			0.949			0.931
Positive	1.000			1.000		
Negative	1.021	00.542–1.922		0.886	0.057–13.698	
HR			0.854			0.906
Positive	1.000			1.000		
Negative	1.061	0.562–2.005		0.843	0.050–14.302	
Ki-67			0.791			0.884
>30%	1.000			1.000		
≤30%	1.090	0.579–2.051		1.051	0.538–2.054	
Molecular subtype			0.607			0.590
Luminal B/HER2+	1.000			1.000		
Nonluminal/HER2+	1.180	0.628–2.216		0.610	0.101–3.678	
Trastuzumab			*0.005*			*0.004*
Yes	1.000			1.000		
No	0.397	0.209–0.754		0.361	0.180–0.725	

**Table 3:** Hazard ratios for DFS prediction in univariate and multivariate analyses.

	Univariate			Multivariate		
	HR	95% CI	*P* value	HR	95% CI	*P* value
Age (year)			0.731			0.917
≤35	1.000			1.000		
>35	0.809	0.242–2.707		0.926	0.216–3.966	
Menopausal status			0.433			0.128
Premenopausal	1.000			1.000		
Postmenopausal	0.726	0.326–1.616		0.475	0.182–1.238	
cT stage			*0.004*			*0.006*
cT1–2	1.000			1.000		
cT3–4	3.166	1.433–6.995		3.801	1.460–9.894	
cN stage			0.559			0.242
cN0	1.000			1.000		
cN1–3	1.265	0.576–2.776		0.545	0.197–1.509	
Grade			0.090			*0.041*
G1–2	1.000			1.000		
G3	3.488	0.822–14.800		5.165	1.069–24.959	
HR			0.056			0.927
Positive	1.000			1.000		
Negative	2.466	0.977–6.127		0.903	0.101–8.084	
Ki-67			0.981			0.607
>30%	1.000			1.000		
≤30%	1.009	0.458–2.227		1.257	0.526–3.007	
Molecular subtype			*0.014*			0.244
Luminal B/HER2+	1.000			1.000		
Nonluminal/HER2+	2.988	1.248–7.155		3.559	0.421–30.056	
Trastuzumab			*0.047*			0.190
Yes	1.000			1.000		
No	2.961	1.015–8.632		2.218	0.674–7.297	
Strict pCR			0.055			0.062
Yes	1.000			1.000		
No	7.065	0.955–52.241		0.144	0.019–1.101	
Lymph node involved			*0.024*			0.074
0	1.000			1.000		
1–3	1.888	0.714–4.992		1.996	0.639–6.237	
≥4	5.296	1.688–16.612		4.855	1.240–19.004	
Endocrine therapy			0.181			0.259
TAM	1.000			1.000		
AI	1.852	0.522–6.563		3.238	0.783–13.398	
No	2.765	0.917–8.342		2.261	0.585–8.737	

## Data Availability

The data used to support the findings of this study are available from the corresponding author upon request.

## References

[1] Chen W., Zheng R., Baade P. D. (2016). Cancer statistics in China, 2015. *CA: a Cancer Journal for Clinicians*.

[2] Valachis A., Nearchou A., Lind P., Mauri D. (2012). Lapatinib, trastuzumab or the combination added to preoperative chemotherapy for breast cancer: a meta-analysis of randomized evidence. *Breast Cancer Research and Treatment*.

[3] Parkinson B., Viney R., Haas M., Goodall S., Srasuebkul P., Pearson S. A. (2016). Real-world evidence: a comparison of the Australian Herceptin Program and clinical trials of trastuzumab for HER2-positive metastatic breast cancer. *PharmacoEconomics*.

[4] Piccart-Gebhart M. J., Procter M., Leyland-Jones B. (2005). Trastuzumab after adjuvant chemotherapy in HER2-positive breast cancer. *The New England Journal of Medicine*.

[5] Cameron D., Piccart-Gebhart M. J., Gelber R. D. (2017). 11 years' follow-up of trastuzumab after adjuvant chemotherapy in HER2-positive early breast cancer: final analysis of the HERceptin Adjuvant (HERA) trial. *The Lancet*.

[6] Baselga J., Carbonell X., Castañeda-Soto N.-J. (2005). Phase II study of efficacy, safety, and pharmacokinetics of trastuzumab monotherapy administered on a 3-weekly schedule. *Journal of Clinical Oncology*.

[7] Mauri D., Pavlidis N., Ioannidis J. P. (2005). Neoadjuvant versus adjuvant systemic treatment in breast cancer: a meta-analysis. *Journal of the National Cancer Institute*.

[8] Cortazar P., Zhang L., Untch M. (2014). Pathological complete response and long-term clinical benefit in breast cancer: the CTNeoBC pooled analysis. *The Lancet*.

[9] Takada M., Ishiguro H., Nagai S. (2014). Survival of HER2-positive primary breast cancer patients treated by neoadjuvant chemotherapy plus trastuzumab: a multicenter retrospective observational study (JBCRG-C03 study). *Breast Cancer Research and Treatment*.

[10] Untch M., Fasching P. A., Konecny G. E. (2011). Pathologic complete response after neoadjuvant chemotherapy plus trastuzumab predicts favorable survival in human epidermal growth factor receptor 2–overexpressing breast cancer: results from the TECHNO trial of the AGO and GBG study groups. *Journal of Clinical Oncology*.

[11] Buzdar A. U., Ibrahim N. K., Francis D. (2005). Significantly higher pathologic complete remission rate after neoadjuvant therapy with trastuzumab, paclitaxel, and epirubicin chemotherapy: results of a randomized trial in human epidermal growth factor receptor 2-positive operable breast cancer. *Journal of Clinical Oncology*.

[12] Gianni L., Eiermann W., Semiglazov V. (2010). Neoadjuvant chemotherapy with trastuzumab followed by adjuvant trastuzumab versus neoadjuvant chemotherapy alone, in patients with HER2-positive locally advanced breast cancer (the NOAH trial): a randomised controlled superiority trial with a parallel HER2-negative cohort. *The Lancet*.

[13] Valachis A., Mauri D., Polyzos N. P., Chlouverakis G., Mavroudis D., Georgoulias V. (2011). Trastuzumab combined to neoadjuvant chemotherapy in patients with HER2-positive breast cancer: a systematic review and meta-analysis. *The Breast*.

[14] Broglio K. R., Quintana M., Foster M. (2016). Association of pathologic complete response to neoadjuvant therapy in HER2-positive breast cancer with long-term outcomes: a meta-analysis. *JAMA Oncology*.

[15] Lyman G. H., Levine M. (2012). Comparative effectiveness research in oncology: an overview. *Journal of Clinical Oncology*.

[16] Korn E. L., Freidlin B. (2012). Methodology for comparative effectiveness research: potential and limitations. *Journal of Clinical Oncology*.

[17] Hahn O. M., Schilsky R. L. (2012). Randomized controlled trials and comparative effectiveness research. *Journal of Clinical Oncology*.

[18] Gianni L., Eiermann W., Semiglazov V. (2014). Neoadjuvant and adjuvant trastuzumab in patients with HER2-positive locally advanced breast cancer (NOAH): follow-up of a randomised controlled superiority trial with a parallel HER2-negative cohort. *The Lancet Oncology*.

[19] Costa R., Kurra G., Greenberg L., Geyer C. (2010). Efficacy and cardiac safety of adjuvant trastuzumab-based chemotherapy regimens for HER2-positive early breast cancer. *Annals of Oncology*.

[20] Gianni L., Pienkowski T., Im Y.-H. (2012). Efficacy and safety of neoadjuvant pertuzumab and trastuzumab in women with locally advanced, inflammatory, or early HER2-positive breast cancer (NeoSphere): a randomised multicentre, open-label, phase 2 trial. *The Lancet Oncology*.

[21] Baselga J., Bradbury I., Eidtmann H. (2012). Lapatinib with trastuzumab for HER2-positive early breast cancer (NeoALTTO): a randomised, open-label, multicentre, phase 3 trial. *The Lancet*.

[22] Peintinger F., Buzdar A. U., Kuerer H. M. (2008). Hormone receptor status and pathologic response of HER2-positive breast cancer treated with neoadjuvant chemotherapy and trastuzumab. *Annals of Oncology*.

[23] Houssami N., Macaskill P., von Minckwitz G., Marinovich M. L., Mamounas E. (2012). Meta-analysis of the association of breast cancer subtype and pathologic complete response to neoadjuvant chemotherapy. *European Journal of Cancer*.

[24] Angelucci D., Tinari N., Grassadonia A. (2013). Long-term outcome of neoadjuvant systemic therapy for locally advanced breast cancer in routine clinical practice. *Journal of Cancer Research and Clinical Oncology*.

[25] Arpino G., Weiss H., Lee A. V. (2005). Estrogen receptor–positive, progesterone receptor–negative breast cancer: association with growth factor receptor expression and tamoxifen resistance. *Journal of the National Cancer Institute*.

[26] Shou J., Massarweh S., Osborne C. K. (2004). Mechanisms of tamoxifen resistance: increased estrogen receptor-HER2/neu cross-talk in ER/HER2–positive breast cancer. *Journal of the National Cancer Institute*.

[27] Montemurro F., Di Cosimo S., Arpino G. (2013). Human epidermal growth factor receptor 2 (HER2)-positive and hormone receptor-positive breast cancer: new insights into molecular interactions and clinical implications. *Annals of Oncology*.

[28] Liu L., Greger J., Shi H. (2009). Novel mechanism of lapatinib resistance in HER2-positive breast tumor cells: activation of AXL. *Cancer Research*.

[29] Xia W., Bacus S., Hegde P. (2006). A model of acquired autoresistance to a potent ErbB2 tyrosine kinase inhibitor and a therapeutic strategy to prevent its onset in breast cancer. *Proceedings of the National Academy of Sciences of the United States of America*.

[30] Wang Y. C., Morrison G., Gillihan R. (2011). Different mechanisms for resistance to trastuzumab versus lapatinib in HER2-positive breast cancers-role of estrogen receptor and HER2 reactivation. *Breast Cancer Research*.

[31] Loibl S., Von Minckwitz G., Schneeweiss A. (2014). PIK3CA mutations are associated with lower rates of pathologic complete response to anti-human epidermal growth factor receptor 2 (her2) therapy in primary HER2-overexpressing breast cancer. *Journal of Clinical Oncology*.

[32] Loibl S., Majewski I., Guarneri V. (2016). *PIK3CA* mutations are associated with reduced pathological complete response rates in primary HER2-positive breast cancer: pooled analysis of 967 patients from five prospective trials investigating lapatinib and trastuzumab^†^. *Annals of Oncology*.

[33] Berns K., Horlings H. M., Hennessy B. T. (2007). A functional genetic approach identifies the PI3K pathway as a major determinant of trastuzumab resistance in breast cancer. *Cancer Cell*.

[34] Miller T. W., Rexer B. N., Garrett J. T., Arteaga C. L. (2011). Mutations in the phosphatidylinositol 3-kinase pathway: role in tumor progression and therapeutic implications in breast cancer. *Breast Cancer Research*.

[35] Ellis H., Ma C. X. (2019). PI3K inhibitors in breast cancer therapy. *Current Oncology Reports*.

[36] Hanker A. B., Pfefferle A. D., Balko J. M. (2013). Mutant *PIK3CA* accelerates HER2-driven transgenic mammary tumors and induces resistance to combinations of anti-HER2 therapies. *Proceedings of the National Academy of Sciences of the United States of America*.

[37] Von Minckwitz G., Untch M., Blohmer J. U. (2012). Definition and impact of pathologic complete response on prognosis after neoadjuvant chemotherapy in various intrinsic breast cancer subtypes. *Journal of Clinical Oncology*.

[38] Kim M., Allen P., Gonzalez-Angulo A. (2013). Pathologic complete response to neoadjuvant chemotherapy with trastuzumab predicts for improved survival in women with HER2-overexpressing breast cancer. *Annals of Oncology*.

[39] Tanioka M., Sasaki M., Shimomura A. (2014). Pathologic complete response after neoadjuvant chemotherapy in HER2-overexpressing breast cancer according to hormonal receptor status. *The Breast*.

[40] Korn E., Sachs M., McShane L. (2015). Statistical controversies in clinical research: assessing pathologic complete response as a trial-level surrogate end point for early-stage breast cancer. *Annals of Oncology*.

[41] Fiteni F., Bonnetain F. (2016). Surrogate end points for overall survival in breast cancer trials: a review. *The Breast*.

[42] Wang R. X., Chen S., Jin X., Chen C. M., Shao Z. M. (2017). Weekly paclitaxel plus carboplatin with or without trastuzumab as neoadjuvant chemotherapy for HER2-positive breast cancer: loss of HER2 amplification and its impact on response and prognosis. *Breast Cancer Research and Treatment*.

